The article "A Fused Multidimensional EEG Classification Method Based on an Extreme Tree Feature Selection" was published in 2022. Journal: Comput Intell Neurosci.

# A Fused Multidimensional EEG Classification Method Based on an Extreme Tree Feature Selection

**DOI:** 10.1155/2022/7609196

**Published:** 2022-08-08

**Authors:** Ruijing Lin, Chaoyi Dong, Pengfei Ma, Shuang Ma, Xiaoyan Chen, Huanzi Liu

**Affiliations:** ^1^College of Electric Power, Inner Mongolia University of Technology, Hohhot 0100801, China; ^2^Intelligent Energy Technology and Equipment Engineering Research Centre of Colleges and Universities in Inner Mongolia Autonomous Region, Inner Mongolia, Hohhot 010051, China

## Abstract

When a brain-computer interface (BCI) is designed, high classification accuracy is difficult to obtain for motor imagery (MI) electroencephalogram (EEG) signals in view of their relatively low signal-to-noise ratio. In this paper, a fused multidimensional classification method based on extreme tree feature selection (FMCM-ETFS) is proposed for discerning motor imagery EEG tasks. First, the EEG signal was filtered by a Butterworth filter for preprocessing. Second, C3, C4, and CZ channels were selected to extract time-frequency domain and spatial domain features using autoregressive (AR), common spatial pattern (CSP), and discrete wavelet transform (DWT). The extracted features were fused for a further feature elimination. Then, the features were selected using three feature selection methods: recursive feature elimination (RFE), principal component analysis method (PCA), and extreme trees (ET). The selected feature vectors were classified using support vector machines (SVM). Finally, a total of twelve subjects' EEG data from Inner Mongolia University of Technology (IMUT data), the 2nd BCI competition in 2003, and the 4th BCI competition in 2008 were employed to show the effectiveness of this proposed FMCM-ETFS method. The results show that the classification accuracy using the multidimensional fused feature extraction (AR + CSP + DWT) is 3%–20% higher than those using the aforementioned three single feature extractions (AR, CSP, and DWT). Extreme trees (ET), which is a sort of tree-based model method, outperforms RFE and PCA by 1%–9% in term of classification accuracies, when these three methods were applied to the procedure of feature extraction, respectively.

## 1. Introduction

As a new method of human-computer interaction, brain-computer interface (BCI) no longer relies on the output pathways of conventional peripheral cerebral nerve and muscle systems but directly uses peripheral auxiliary devices such as sensors, amplifiers, and computers to collect and analyze electroencephalogram (EEG) signals [1, 2]. Thus, the action intentions contained in brains can be extracted and deciphered for the purpose of information interaction between brains and the outside world [3]. Motor imagery (MI), as a typical BCI, refers to the act of imagining a specific action but not actually performing that action, and has received widespread attention in fields such as neuroscience and artificial intelligence [4, 5].

The EEG signals of different MI tasks are usually accompanied by different sensory-motor rhythm (SMR), i.e., increased and decreased power in specific frequency bands in various brain regions, and mathematical feature vectors can be extracted from the SMR using a feature extraction algorithm and fed into a classifier for classification [6, 7]. The classical feature extraction method on the time domain is the autoregressive (AR). Wang and Chen used a hierarchical vector AR [8], and Liu et al. proposed a feature extraction method based on the combination of phase synchronization and AR model coefficients [9]. These two feature extraction methods mainly focused on the feature extractions in the time domain and obtained a satisfactory classification accuracy for the investigated MI tasks [8, 9]. The typical feature extraction method in the time-frequency domain is the wavelet transform (WT). WT can characterize EEG signals in both time and frequency domains and decompose these EEG signals into multiple frequency bands to reveal different time-frequency features. Nevertheless, WT relies heavily on a priori knowledge to extract the frequency bands of interest [10]. This fact limits the application scope of WT. In another aspect, the common spatial pattern (CSP) extracts the features reflecting the different power distributions in the spatial domain for different MI tasks. Later, researchers combined CSP with other optimization algorithms or classification methods to improve its performance in classification accuracy. For example, Feng et al. proposed a new correlation-based time window selection (CTWS) algorithm [11]. The algorithm used correlation analysis to select an optimal reference signal and the starting point of time windows for each class, so that the average classification accuracy of MI-based BCI was substantially improved in combination with the traditional CSP. Bao Liu et al. proposed a PSO-CSP-SVM that was applied to MI feature extraction [12]. Gu et al. combined CSP with a convolutional neural network (CNN) to extract high-level characteristics of original data [13]. Pei et al. considered that the CSP algorithm usually cannot extract adequate frequency band features [14]. To overcome this shortcoming of the CSP, the paper proposed a tensor-based frequency feature combination (TFFC) method to construct a new feature set by fusing broadband features with narrowband features. Thus, the dependence on a classifier can be reduced and the adaptiveness of the features can be increased.

Each of the aforementioned methods has its own advantages, but they also have limitations when they are applied to further improve the classification accuracy of MI tasks in fact. These methods only consider some partial aspects of features underlying MI EEG signals and cannot fully reflect data characteristics and network information flows. This paper proposes a fused multidimensional classification method based on extreme tree feature selection (FMCM-ETFS) in classifying motor imagery (MI) EEG signals. The specific process is as follows: First, the EEG signals are filtered by a Butterworth filter to obtain a purified EEG signal. Second, AR, CSP, and DWT are used to extract the AR model coefficients, the variance and mean after CSP filtering, and the wavelet coefficients. These three methods can effectively extract time, frequency, and spatial domain features of EEG signals together to meet the signal dimensional diversity and yield more comprehensive information. Therefore, the three sorts of features were fused to obtain an augmented feature vector including all features. Then, the complexity of the classifier models is further decreased by three feature selection methods according to the support vector machine (SVM) classifier. The three methods are recursive feature elimination (RFE), principal component analysis method (PCA), and extreme tree (ET). Finally, a total of twelve subjects' EEG data from Inner Mongolia University of Technology (IMUT data), the 2nd BCI competition in 2003 [15], and the 4th BCI competition in 2008 [16] are applied to validate the effectiveness of the proposed FMCM-ETFS. The experimental results show that the FMCM combined with ET obtained 1%–9% higher accuracy than the FMCM combined with RFE or PCA on average.

## 2. Feature Extraction Methods

### 2.1. AR Model

The AR model is a fundamental technique in time-series analysis and is widely used in BCI data processing [17]. The definition of the AR model is as follows: if there is a time series {*y*(*t*);  t=1,2,…, *n*} consisting of *n* sample points at an equal time period, the time series can be regressed (or predicted) on its values at multiple previous moments, using the following formula:

(1) $$\begin{array}{c} y\left(t\right)=-\sum_{i=1}^{p}a_{i}y\left(t-i\right)+e\left(t\right), \end{array}$$

where *e*(*t*) is a white noise series with mean 0, *p* is the order of the AR model, and *a*_*i*_ are the coefficients of the AR model [18].

### 2.2. CSP

The CSP algorithm is a spatial domain filtering and feature extraction algorithm for two categories tasks, capable of extracting the spatially distributed characteristics of each class from multi-channel EEG signals. The basic principle of CSP algorithm is to find a set of optimal spatial filters for yielding a projection. This projection uses matrix diagonalization to maximize the difference between the variances of the two categorical signals, thus obtaining feature vectors with a high degree of discrimination [19].

The experimentally measured EEG data is represented as an *M* × *N* matrix *X*, where *M* is the number of channels and *N* is the number of sampling points per channel [20]. Using *R*_1_ and *R*_2_ to denote the normalized covariance matrices of the left-handed motion imagery and the right-handed motion imagery. Then, a normalized covariance matrix of EEG data is as follows:

(2) $$\begin{array}{c} R_{1}=\frac{X_{1}X_{1}{}^{T}}{\text{trace}X_{1}X_{1}{}^{T}},\\ R_{2}=\frac{X_{2}X_{2}{}^{T}}{\text{trace}X_{2}X_{2}{}^{T}}. \end{array}$$

Respectively, the mixed-space covariance matrix can be represented as follows:

(3) $$\begin{array}{c} R_{m}=\bar{R_{1}}+\bar{R_{2}}. \end{array}$$

An eigenvalue decomposition is carried out according to the mixed space covariance matrix by the following equation(4):

(4) $$\begin{array}{c} R_{m}=U\lambda U^{T}, \end{array}$$

where matrix *λ* is the diagonal matrix with the eigenvalues of *R*_*m*_ and *U* is the corresponding eigenvector matrix of *λ*. Thus, the whitened matrix *P* of *R*_*m*_ is derived as follows:

(5) $$\begin{array}{c} P=\sqrt{\lambda^{-1}}U^{T}. \end{array}$$

Then, two transformations of *R*_1_ and *R*_2_ is performed as follows :

(6) $$\begin{array}{c} S_{1}=PR_{1}P^{T},\\ S_{2}=PR_{2}P^{T}. \end{array}$$

After principal component decompositions of *S*_1_ and *S*_2_, it can be proved that the eigenvector matrices of *S*_1_ and *S*_2_ are equal, and the sum of *λ*_1_ and *λ*_2_ is the identity matrix. Thus, the spatial filter *W* is constructed as follows:

(7) $$\begin{array}{c} W=B^{T}P, \end{array}$$

where *B* is the eigenvector matrix of *S*_1_ and *S*_2_.

### 2.3. DWT

WT is a transform analysis method, inheriting and developing the idea of localization in a short-time Fourier transform. As an ideal tool for the time-frequency analysis of signals, WT overcomes the shortcoming that the time-frequency window is fixed and cannot be adjusted with frequency [21]. The continuous wavelet transform (CWT) is defined as follows:

(8) $$\begin{array}{c} W_{x}\left(a,b\right)={\left|a\right|}^{-1/2}\int x\left(t\right)\psi \left(\frac{t-b}{a}\right)\text{d}t=\langle x\left(t\right),\psi_{a,b}\left(t\right)\rangle , \end{array}$$

where *ψ*_*a*,*b*_(*t*)=|*a*|^−1/2^*ψ*(*t* − *b*/*a*) is a wavelet function. The parameter *a* is the scaling factor of the wavelet function, and *b* is the translation parameter of the wavelet function. The two parameters adjust the frequency scale and the time scale, respectively. The subsequent wavelet transforms of the same signal can vary for different mother wavelets. The discrete wavelet transform (DWT) requires the discretization of CWT:

(9) $$\begin{array}{c} W_{x}\left(j,r\right)=2^{-j/2}\int x\left(t\right)\psi \left(2^{-j}t-r\right)\text{d}t=\langle x\left(t\right),\psi_{j,r}\left(t\right)\rangle , \end{array}$$

where Ψ_*j*,*r*_(*t*)=2^−*j*/2^Ψ(2^−*j*^*t* − *r*) is called a dyadic wavelet.

## 3. Feature Selection Methods

### 3.1. Recursive Feature Elimination

RFE works by searching a subset of features starting from all features of the training data and successfully removing features until a desired number of features are retained in performing classifications by SVM [22]. This is achieved by fitting a given mathematical model, ranking the features by their importance, discarding unimportant features, and refitting the model recursively. This process is repeated until a specific number of features are retained [23]. The description of the RFE algorithm is described as follows:

(1) The training samples are *x*={*x*_1_, *x*_2_,…,*x*_*k*_,…,*x*_*n*_}^*T*^. The class labels are *y*={*y*_1_, *y*_2_,…,*y*_*k*_,…,*y*_*n*_}^*T*^. External estimators are selected as the basis of constructing an SVM.
(2) The estimators are trained using the squared weight coefficients *w*^2^ as the feature importance criterion. The formula for the weight vector is as follows:
  (10) $$\begin{array}{c} w=\sum_{k}\alpha_{k}y_{k}x_{k}, \end{array}$$
where *α*_*k*_ is the Lagrange multiplier.
(3) The feature weight values are ranked and the features with the smallest contribution are removed, one feature at a time.
(4) Steps 2 and 3 are repeated until the number of features reaches a specified threshold.

### 3.2. Principal Component Analysis

The main purpose of PCA is to explain most of the variation in the original data with fewer variables by transforming many highly correlated variables into variables that are uncorrelated with each other [24]. Usually, a few new variables, called principal components, are selected to explain most of the variation in the data instead of using all the original variables. PCA attempts to reduce the dimensionality of the original variable space, simultaneously losing less information as possible. The detailed procedure of PCA was surveyed in [25].

### 3.3. Tree-Based Model

As a sort of embedded feature filtering algorithm, tree-based model algorithms are based on machine learning theory to analyze the importance of features, so the most important feature can be preserved and selected. Random forests (RF) and extreme trees (ET) are two sorts of typical tree-based model algorithms.

RF is an integrated learning method based on bagging method, and the advantage of this integrated algorithm is that each decision tree is constructed by random variables [26]. The randomness of RF lies in: sample randomization, feature randomization, parameter randomization, and model randomization. ET is a variant of the RF algorithm with a different stochastic process [27]. ET uses all training samples as training samples to build each decision tree, and randomly draws segmentation rules on each node to select the optimal segmentation rules by scores [26]. Therefore, another characteristic of randomness, i.e., split randomness, is introduced. This spilt randomness greatly enhances the independence between each decision tree, thus, it improves the training speed and generalization ability of the classifiers. ET algorithm is described as follows:

(1) All original *D* training samples are selected as training data input.
(2) A decision tree is constructed from *m* features {*f*_1_, *f*_2_,…, *f*_*m*_} randomly selected from the whole *M* features without replacement. In general, *m* is smaller than or equal to *M.*
(3) The division values {*d*_1_, *d*_2_,…, *d*_*m*_} are randomly selected between their maximum and minimum values for each of these *m* features sequentially, and the optimal split value *d*_*j*_(*j*=1,2,…, *m*) is selected by a particular normalization of the information gain. The formula for the particular normalization of the information gain is as follows:
  (11) $$\begin{array}{c} {\text{Score}}_{C}\left(d,D\right)=\frac{2I_{C}^{d}\left(D\right)}{H_{d}\left(D\right)+H_{C}\left(D\right)}, \end{array}$$
where *H*_*C*_(*D*) is the (log) entropy of the classification in *D*, *H*_*d*_(*D*) is the split entropy, and *I*_*C*_^*d*^(*D*) is the mutual information of the split outcome and the classification [27].
(4) Steps 2 and 3 are repeated until the multiple decision trees are constructed to obtain an extreme forest.

## 4. Algorithm Structure of FMCM-ETFS

### 4.1. Overview of FMCM-ETFS Algorithm Structure

The proposed FMCM-ETFS includes two procedures: 1. The experiment procedure collecting MI EEG dataset from IMUT (6 subjects) or the direct use of dataset III from the 2nd BCI competition 2003 (1 subject) and dataset 2b from the 4th BCI competition 2008 (5 subjects); 2. The data processing procedure consisting of data processing, feature extraction, feature selection, and pattern classification. A scheme of FMCM-ETFS is shown in Figure 1. For the data preprocessing, the collected EEG signals are band-pass filtered by a Butterworth filter since most of the response frequency band of MI EEG signal is 8–30 Hz. Therefore, the passband frequency of the filter is set at 8–30 Hz. At the same time, the order of the filter is set at 4. For the feature extraction, three methods: AR, CSP, and DWT, are used to obtain the features of EEG signals both in the time-frequency domain and the spatial domain. Then, all the extracted features are fused to obtain a whole feature vector. In the subsequent feature extraction, the fused features are selected by three methods: RFE, PCA, and ET to obtain the optimal subset of features and eliminate irrelevant and redundant features. Finally, the screened features are classified by a SVM, and the performance of the three feature selection methods is compared in terms of classification accuracy.

### 4.2. Feature Fusion Method

MI EEG signals always include complex and diverse information from various brain regions. However, extracting features from one dimension alone does not reflect this comprehensive information. Therefore, this paper uses a feature fusion algorithm to obtain fused features in time, frequency, and spatial domains, which represent three-dimensional characteristics of brain networks. First, the coefficients of the AR model are extracted by the AR algorithm to construct a feature vector, so the time-domain features of the EEG signals can be obtained initially. Second, the spatial domain features of the EEG signals are obtained by CSP with the variance of each channel as the feature vector. Finally, the time-frequency domain features of the EEG signals were extracted by DWT using Daubechies class db4 wavelets for 3-layer decomposition, and the mean value of the squared coefficients in layer 3 of each channel was used as the feature vector.

### 4.3. Feature Selection Method

The fused features usually have some irrelevant and redundant features while the information content accumulates. This makes the classification model too complex and overfitted, which causes the prediction accuracy to decrease. To address this difficulty, this paper adopts three feature selection algorithms: RFE, PCA, and ET, to screen the fused features and reduce the dimensionality of the features while ensuring the necessary information content of the features is preserved.

REF uses a support vector regression (SVR) model to train the EEG data and removes one feature at a time, which is based on the weight coefficients in the models, until 20 features are left. In PCA, the number of principal components is set at 20, and then dimensionality reduction on the fused features is performed subsequently. The last applied approach is ET, which is a sort of tree-based model algorithm. The performance of ET depends on the adjustment of three parameters, i.e. *m*, *n*_min_, and R. The notation *m* denotes the total number of randomly selected features for each node, which is usually set to $\sqrt{M}$. The notation *M* denotes the total number of features. This default setting has proven to be the optimal way to solve various problems [27]. The notation *n*_min_ represents the minimum sample size for the splitting nodes. Smaller values of *n*_min_ result in deeper forests, and in this paper *n*_min_=2 is used as a default value. *R* denotes the number of trees. In practice, the larger the value of *R* is, the higher the accuracy can be arrived [24]. However, a large tree number usually causes the algorithm difficult to converge. In this paper, *R* is at 10. Finally, the classification accuracies of the three feature elimination methods are compared to determine the choice of elimination methods.

### 4.4. Classification Algorithm

There are four kernel functions, for examples, linear kernel, polynomial kernel, Sigmoid kernel, and radial basis kernel, commonly used to construct different classifiers in SVM methods [28]. In this paper, the following linear kernel function is used:

(12) $$\begin{array}{c} k\left(x_{i},x_{j}\right)=x_{i}\cdot x_{j}, \end{array}$$

where *x*_*i*_ and *x*_*j*_ denote the *i*-th and *j*-th samples, respectively. For the SVM classifier, the error penalty factor *C* is a major parameter that affects the performance of the SVM classifier. The parameter is determined by a grid search and validated by a 10-fold cross-validation.

## 5. Experiment

### 5.1. Experimental Data Set

The dataset used in this paper comes from three sources: 1. MI EEG dataset III in 2003 BCI competition from Graz University of Technology; 2. MI EEG dataset 2b in 2008 BCI competition from Graz University of Technology; 3. EEG dataset from Inner Mongolia University of Technology (IMUT data) recoded by a 32-channel EEG acquisition device from Brain Products (BP) Inc., Germany.

The 2003 BCI competition dataset III contains 7 sets of experiments with 40 trials for each set of experiments, totally yielding 280 trials of MI data. The EEG acquisition device consisted of a G.tec amplifier and Ag/AgCl electrodes to acquire EEG data with a sampling frequency of 128 Hz, and the EEG data of 3 channels namely C3, C4, and Cz were recorded. The experimental data were divided into two parts, i.e., the training set and the testing set, each of which included 140 trials of experiments (70 experiments for left-handed MI and 70 experiments for right-handed MI).

The 2008 BCI competition dataset 2b contains 6 runs with ten trials per run. Each subject participated in two screening sessions without feedback, recorded on two different days within two weeks. This resulted in 20 trials per run and 120 trials per session. Data of 240 repetitions of each MI class were available for each subject in total. An EEG acquisition device acquires the EEG data with a sampling frequency of 250 Hz, and the EEG data of 3 channels C3, C4, and Cz were recorded.

The data from IMUT were collected using a 32-channel EEG acquisition device from BP Inc. at a sampling frequency of 500 Hz. The subjects include six males around 25 years of age, and the experiments were conducted in a quiet environment. The experimental timing diagram is shown in Figure 2. At the beginning of the experiment (*t* = 0 s), the screen was black and the subject remained at rest; two seconds later, the screen appeared a “+”cross, prompting the subject to get ready; one second later, the screen appeared a left or right arrow lasting 6 s prompting the subject to start MI of the left or right hand. A total of 80 experiments were performed for each set of experimental data, including 40 left-handed MI experiments and 40 right-handed MI experiments. The details of the data are shown in Table 1.

### 5.2. Experimental Results

Table 2 provides a comparison of the classification accuracies between using AR features, CSP features, DWT features, and AR + CSP + DWT features, which reflect the multidimensional fused features for the laboratory-collected IMUT data. The accuracy of using AR + CSP + DWT features is on average 14.1% higher than that of using AR features, 15.5% higher than that of using CSP features, and 16.9% higher than that of using DWT features. The datasets III BCI 2003 and 2b BCI 2008 also validates a similar trend that the average classification accuracy using AR + CSP + DWT features is higher than the average classification accuracy using a single category of features. The results for the two public datasets are presented in Table 3. The accuracy of using AR + CSP + DWT features is on average 18.5% higher than that of using AR features, 15% higher than that of using CSP features, and 11.1% higher than that of using DWT features. We have deleted the feature categories one by one in the sequence of AR, CSP, and DWT. For IMUT data, the average classification accuracies are as follows: 0.707 for CSP + DWT + SVM, 0.717 for AR + DWT + SVM, and 0.754 for AR + CSP + SVM (see Table 2). Compared to AR + CSP + DWT + SVM, CSP + DWT + SVM shows a decrease of 0.068, which is the largest decrease magnitude among the other two decreases of CSP + DWT + SVM and AR + DWT + SVM. Therefore, the feature category of AR contributes most to the proposed AR + CSP + DWT + SVM in terms of classification accuracy. The same conclusion can also be obtained for datasets III BCI 2003 and 2b BCI 2008 (see Table 3).

Table 4 shows a comparison of the classification accuracies using three feature selection algorithms (RFE, PCA, and ET) for the laboratory-collected IMUT data. ET works better than REF and PCA because the classification accuracy of ET + SVM is on average 3.3% (*p* = 0.0346 <0.05, *t*-test) higher than that of RFE + SVM and 2.68% (*p* = 8.9771e-4 <0.01, *t*-test) higher than that of PCA + SVM. A similar trend also applied to the datasets III BCI 2003 and 2b BCI 2008. The experimental results are demonstrated in Table 5, where ET + SVM outperforms 3.5% (*p* = 0.014 <0.05, *t*-test) than RFE + SVM and 3.65% (*p* = 0.0014 <0.01, *t*-test) higher than PCA + SVM. The advantage of feature selections also is shown in Figures 3 and 4. Figures 3 and 4 show a comparison of the classification accuracy with and without the feature selection algorithm under the IMUT data, datasets III BCI 2003 and 2b BCI 2008, respectively. In Figures 3 and 4, the classification accuracy using the fused features selected by ET is significantly higher than that using the fused features without any feature selection. F_feature represents using the fused features without any selection. RFE_F_feature represents using the fused features with RFE model selection, PCA_F_feature represents using the fused features with PCA selection, and ET_F_feature represents using the fused features with ET model selection. A similar situation also happened when using RFE and PCA as feature selection methods.

To further verify the effectiveness of the proposed FMCM-ETFS, another feature selection algorithm ReliefF proposed in the literature [29], was selected to compare with the ET feature selection method. The comparison result is detailed in Figure 5, where the average classification accuracy of the ET + SVM algorithm for IMUT data is 2.43% (*p* = 0.0029 <0.01, *t*-test) higher than that of ReliefF + SVM algorithm (see Figure 5(a)). The same trend retains in datasets III BCI 2003 and 2b BCI 2008, where the average classification accuracy of the ET + SVM algorithm was 2.99% (*p* = 0.0061 <0.01, *t*-test) higher than that of the ReliefF + SVM algorithm (see Figure 5(b)).

## 6. Conclusion

In this paper, we propose a fused multidimensional classification method based on extreme tree feature selection in the task of discerning MI EEG. The fused multidimensional features include the features extracted by AR, CSP, and DWT algorithms that reflect the complex information of MI EEG signals from various dimensions: time, frequency, and space domain. Furthermore, to avoid the overfitted model problem, three feature selection methods, RFE, PCA, and ET are applied to lower the complexity of the machine learning models. The experiment results for the datasets from IMUT and Graz University show that the accuracy of using AR + CSP + DWT features is 3%–23% higher than that of using the single-dimensional features and ET has 3%–4% higher accuracy than the other two feature selection algorithms. This result of the study convergingly verifies that a fused multidimensional classification method based on extreme tree feature selection (FMCM-ETFS) can significantly improve the performance of the MI EEG classifiers.

## Figures and Tables

**Figure 1:** Scheme of FMCM-ETFS.

**Figure 2:** Experimental timing diagram of IMUT EEG data recording.

**Figure 3:** The comparison of classification accuracies with feature selection and without any feature selections for IMUT data. (a) Before and after RFE; (b) before and after PCA; (c) before and after ET.

**Figure 4:** The comparison of classification accuracies with feature selection and without any feature selections for datasets III BCI 2003 and 2b BCI 2008. (a) Before and after RFE; (b) before and after PCA; (c) before and after ET.

**Figure 5:** Comparison of classification accuracies between ET and ReliefF for IMUT data, datasets III BCI 2003 and 2b BCI 2008. (a) IMUT data; (b) datasets III BCI 2003 and 2b BCI 2008.

**Table 1:** The statistics of experimental datasets from IMUT and BCI competitions (Graz University of Technology).

Dataset	Experimental dataset	Public datasets	
	IMUT data	III BCI 2003	2b BCI 2008
Number of subjects	6	1	5
Number of channels	3	3	3
Number of experiments (times/person)	80	280	240

**Table 2:** Classification accuracy for IMUT data using different feature extraction methods.

Dataset	Experimental dataset					
	IMUT data					
	*a*	*b*	*c*	*d*	*e*	*f*
AR + SVM	0.660	0.641	0.575	0.486	0.720	0.721
CSP + SVM	0.638	0.567	0.656	0.569	0.511	0.778
DWT + SVM	0.558	0.630	0.498	0.518	0.650	0.780
CSP + DWT + SVM	0.613	0.763	0.825	0.613	0.625	0.800
AR + DWT + SVM	0.725	0.800	0.513	0.600	0.825	0.838
AR + CSP + SVM	0.675	0.850	0.788	0.525	0.813	0.875
AR + CSP + DWT + SVM	**0.700**	**0.837**	**0.812**	**0.600**	**0.825**	**0.875**

**Table 3:** Classification accuracy for datasets III BCI 2003 and 2b BCI 2008 using different feature extraction methods.

Dataset	Public datasets					
	III BCI 2003			2b BCI 2008		
	aa	bb	cc	dd	ee	ff
AR + SVM	0.622	0.416	0.397	0.649	0.551	0.596
CSP + SVM	0.420	0.493	0.580	0.786	0.541	0.622
DWT + SVM	0.451	0.573	0.668	0.742	0.657	0.585
DWT + CSP + SVM	0.693	0.659	0.775	0.808	0.617	0.658
AR + DWT + SVM	0.636	0.725	0.667	0.792	0.758	0.700
AR + CSP + SVM	0.650	0.783	0.633	0.808	0.683	0.675
AR + CSP + DWT + SVM	**0.650**	**0.725**	**0.742**	**0.817**	**0.733**	**0.675**

**Table 4:** Classification accuracy for IMUT data of using different feature selection methods.

Dataset	Experimental dataset					
	IMUT data					
	*a*	*b*	*c*	*d*	*e*	*f*
RFE + SVM	0.700	0.850	0.775	0.600	0.825	0.875
PCA + SVM	0.700	0.837	0.825	0.600	0.825	0.875
ET + SVM	**0.737**	**0.862**	**0.862**	**0.625**	**0.850**	**0.887**

**Table 5:** Classification accuracy for datasets III BCI 2003 and 2b BCI 2008 using different feature selection methods.

Dataset	Public datasets					
	III BCI 2003			2b BCI 2008		
	aa	bb	cc	dd	ee	ff
RFE + SVM	0.650	0.750	0.742	0.833	0.675	0.708
PCA + SVM	0.664	0.725	0.742	0.808	0.733	0.675
**ET** **+** **SVM**	**0.692**	**0.783**	**0.775**	**0.850**	**0.750**	**0.717**

## Data Availability

The data used to support the findings of this study are available from the corresponding author upon request.
